# The Efficacy of Acupuncture on Patients with Erectile Dysfunction: A Review

**DOI:** 10.1155/2022/4807271

**Published:** 2022-05-09

**Authors:** Hao Wang, Ming Zhao, Jiwei Zhang, Bin Yan, Shengjing Liu, Feng Zhao, Jun Guo, Fu Wang

**Affiliations:** Department of Andrology, Xiyuan Hospital of China Academy of Chinese Medical Sciences, 1 Caochang, Xiyuan, Beijing 100091, China

## Abstract

Erectile dysfunction (ED) is one of the most common sexual dysfunctions in men. The prevalence of ED has been increasing in recent years, which has critically affected male reproductive health and quality of life. According to various guidelines, phosphodiesterase-5 inhibitors are the most commonly recommended drugs for treating ED. However, many patients turn to alternative therapies because of adverse reactions, such as headache, and the poor efficacy of these drugs. Acupuncture is a long-established treatment in traditional Chinese medicine (TCM) and has been approved by the World Health Organization for improving penile erection as well as other discomforts in patients. However, previous systematic reviews have not discussed the characteristics and the related mechanisms of acupuncture treatment. Therefore, this study focuses on summarizing the characteristics and advantages of TCM in acupuncture treatment for ED based on relevant literature and on predicting and analyzing the related mechanisms.

## 1. Introduction

Erectile dysfunction (ED) refers to the condition in which a man cannot achieve or maintain an erection long enough to engage in a satisfying sex life [1]. It is one of the most common sexual dysfunctions among men and can influence mental and physical health, as well as the quality of life. In 2019, Goldstein et al. showed that in the eight countries covered in their study, the average age of men with ED was 51.98 years [2]. Another study observed that the global prevalence rate of ED in men aged 40–70 years was 52% [3], with an upward trend in the future [4, 5]. According to the European Association of Urology (EAU) guidelines on sexual and reproductive health, the treatment for ED involves 9 different options, including oral pharmacotherapy, topical/intraurethral alprostadil, intracavernous injection therapy, and hormonal treatment [6]. These therapies are not always effective and may have adverse effects, such as cardiovascular dysfunction, hearing impairment, penile pain, and numbness [7–9]. Additionally, patients with ED may also suffer from sleep disorders [10], anxiety [11], muscle weakness [12], cold or chills, and other bodily symptoms. The medications can sometimes even increase the risks for sexual dysfunction. Hence, relying only on conventional treatments may cause difficulties in resolving the symptoms. In recent years, an increasing number of scientists and scholars have tried to apply alternative therapies to treat ED, such as acupuncture and Chinese medicine. Acupuncture has especially turned out to be an indicated treatment for ED [13].

Acupuncture is a key component of traditional Chinese medicine (TCM) as it attaches immense importance to the integration of this concept. Acupuncture has been used quite frequently for treating various urologic disorders, including both male and female sexual dysfunctions [14, 15], with a majority of the research focusing on ED [16]. Many systematic reviews have analyzed the current evidence on ED treatment to prove or discuss their effects [17]. However, discussions on the similarities and differences between the treatments are not sufficient. We only understand the effects of these treatments, and the means to achieve these results consistently remain unclear. This aspect of the treatment should be given much more attention. For example, apart from the holistic and macro analysis of clinical trials, related mechanisms, acupuncture points, depths of the needles, and the meridians in which the acupoints are located are also necessary parts of the discussion. Therefore, unlike other systematic reviews, this review focuses on such important aspects and the Chinese or Western medicine theories behind them along with their clinical references.

## 2. Method

### 2.1. Search Strategy

PubMed, EMBASE, and Cochrane Library were searched from October 6, 2021. The search was performed in English. The following search terms were used: acupuncture, acupuncture treatment, electroacupuncture (EA), acupuncture therapy, fire needling, scalp acupuncture, ear acupuncture, ED, impotence, erection failure, penis erection, male sexual dysfunction, clinical trial, clinical study, controlled study, randomized controlled trial, and placebo (Table 1). Relevant citations from the reference list were also used.

### 2.2. Eligibility Criteria

#### 2.2.1. Inclusion Criteria

1. Types of participants: the subjects were patients above the age of 18 years who were diagnosed with ED (both psychological ED and organic ED) using clinical and/or instrumental methods regardless of ethnicity, country, and course.
2. Types of interventions: common acupuncture (including acupuncture, EA, fire needling, scalp acupuncture, and ear acupuncture) alone or combined with other treatment methods were used in the treatment group regardless of the position of the acupoints, treatment frequency, and course. The establishment of a control group was not required.
3. Types of comparisons: the control group underwent conventional treatment, medication, placebo acupuncture, sham acupuncture, or no treatment, or there were no control groups
4. Types of outcomes: international index of erectile function 5 (IIEF 5), effective rate, self-sexual activity, improvement in depression or anxiety, and safety indicators and adverse reactions were included.
5. Types of studies: randomized controlled trials (RCTs), uncontrolled clinical trials (UCTs), and other prospective clinical trials were included, and the qualified papers were limited to the English language.

#### 2.2.2. Exclusion Criteria

1. Patients with external genital malformation or organic damage to the genitourinary system (such as a pudendal nerve injury from trauma or surgery).
2. Nonclinical studies, review articles, animal experiments, case series, case reports, and cross-over studies
3. Nonacupuncture therapy, including moxibustion, acupoint application, and massage of the related acupoints
4. Duplicate publications and trials with incomplete data.

### 2.3. Data Collection and Analysis

#### 2.3.1. Selection of Studies

The two authors (Hao Wang and Ming Zhao) searched the articles according to the outline retrieval strategy and summarized the results. Duplicate literature were removed, some literature were excluded after analyzing the content of the title and abstract, and literature that did not meet the inclusion and exclusion criteria were removed after analysis of the full text. Dissenting opinions were submitted to another author (Bin Yan) for adjudication throughout the whole process (Figure 1).

#### 2.3.2. Data Extraction

The data were extracted independently by two authors (Hao Wang and Ming Zhao) in a standard form. The extracted contents included author, publication date, study design, type of ED, number of participants treated using acupuncture, acupuncture points, types of acupuncture therapy, duration of the session, types of outcomes measured, reported outcomes, and adverse events (Table 2). The extracted data were compared by two authors to ensure accuracy and completeness. Another author (Bin Yan) participated in discussions and resolved any disagreements.

## 3. Result

According to the above screening process, there were 4 English-language, human clinical trials on acupuncture for treating ED, including two RCTs and two UCTs. 70 of them were treated with acupuncture. Three of these studies included nonorganic ED, including two marked as psychological ED. The remaining study included nine patients with psychological ED and four with organic ED. The acupuncture points and interventions were different. In Engelhardt's study [18], 21 subjects were randomized to acupuncture (10) and placebo acupuncture (11) groups. In the placebo group, the acupuncture points that were used were the ones to treat headache (Xuan Zhong (GB39), Jie Xi (ST41), and Tian Shu (ST25)). Each acupuncture session lasted 20 minutes, with 1 to 2 sessions per week, ranging from 5 to 20 sessions, with 20 sessions considered to be the maximum number of treatments. Completed by two certified acupuncturists, the treatments were considered effective when an erection was achieved that was sufficient for penetration and sexual intercourse. On average, after 6.2 acupuncture sessions (range: 4–10) in 11 cases of the placebo acupuncture group, there was only 1 patient with improvement seen. According to the protocol, the other 10 patients with no improvement in the sham acupuncture group were crossed over to the acupuncture group. Ultimately, a total of 19 patients in the acupuncture group completed the acupuncture treatment (1 lost to follow-up), and 13 of them improved. In Aydin's trial [19], 15 cases in the acupuncture group were subjected to a 3 Hz direct current to produce electrical stimulation after the insertion of the needles, which boosted the effect of the acupuncture needles. Each treatment lasted 20 minutes and occurred twice a week for 6 weeks, however, the specific manipulations utilized were not mentioned. Fourteen cases of the placebo acupuncture group were selected for nontraditional acupuncture points that were different from the acupuncture group, and EA was added. However, the specific locations and depths of acupuncture were not mentioned. In the acupuncture group, 9 of the 15 patients showed significant improvement after six weeks of treatment, with an overall response rate of 60%, and 6 patients in the placebo acupuncture group showed significant improvement, with an overall response rate of 43%. As in the case of Engelhardt's study, it is not clear how the acupuncture was specifically performed and whether blindness was used. In Kho's study [20], 16 subjects were treated with 8 sessions of acupuncture twice a week for 4 weeks. Eight acupoints were acupunctured in each session. After achieving qi, low-frequency electrical stimulation (5 Hz, 10 mA) was performed at Guan Yuan (CV4), Bai Hui (GV20), and San Yinjiao (SP6) on both sides for 30 minutes. To assess the changes in the concentration of stress hormones, blood samples were drawn according to a fixed time schedule. After treatment, two patients achieved a better erection (15%), and four patients demonstrated an increase in sexual activity (31%). The final interview also revealed that 2 months after the first treatment, five patients continued to experience improvement in their sex life in terms of activity and overall quality of erection (39%). The overall improvement rate was 54% (7 out of 13 patients). In Yaman's trial [21], 29 patients with ED without organic lesions were selected, and acupuncture needles of different lengths were selected in different clinical operations at different sites. The needles were retained for 20 minutes after de qi. All patients received acupuncture three times in the first week, followed by two times a week for a fixed course of 10 times, as well as another 10 courses of acupuncture if the treatment failed. The treatment was deemed effective if the patient had sex two or more times a week. After acupuncture treatment, 20 patients (69%) responded to the treatment, whereas 9 patients (31%) did not. Premature ejaculation was observed in two of the nine unsuccessful cases.

Although the acupoints selected in the four studies were different, they also had certain commonalities. Statistical analysis was performed on the frequency of the acupuncture points involved in each study. It was found that the acupuncture points were chiefly located on the distal extremities (9/24) and abdomen (7/24). The meridians of the acupoints were mainly CV (6/24) and KI (4/24). In terms of outcome indicators, all the studies used self-reported sexual activities, with one study adding IIEF 5 and another utilizing partner satisfaction and the profile of hormones as well. All the studies showed that acupuncture had beneficial effects on ED, with effective rates from 54% to 69%. Only the one study that included organic ED patients showed an improvement in sexual activity. Engelhaedt et al. confirmed its positive influence using IIEF5 as an indicator, and another study by Kho et al. proved no significant change in sex hormone levels and partner satisfaction.

## 4. Discussion

### 4.1. Characteristics and Treatment of TCM

Although PDE5Is have resulted in significant progress when it comes to ED treatment, Carvalheira et al.'s study showed that after years of treatment, the effective rate was difficult to further improve and that there was a high rate of treatment failure and termination [22]. Furthermore, evidence shows that 20% to 30% of patients treated with orally-administered PDE5Is exhibit no significant effect [23]. The reasons for this lack of effect may include diabetes, hypertension, or pelvic trauma. However, a high percentage of the patients in the clinic were young adults who suffered from none of these conditions [24, 25]. Some men may achieve an adequate erection for intercourse but eventually discontinue the medication owing to unrealistic expectations or low acceptance, such as inadequate knowledge of the therapeutic nature of the drug or mistakenly considering it as an aphrodisiac [26].

In China, acupuncture is an irreplaceable traditional treatment method and has been passed down for more than two thousand years. Acupuncture has a broad basis of practice and has been recognized and accepted by the Chinese people. The purpose of the therapy is to relieve the patients' symptoms via a holistic approach, according to the 2010 European Association of Urology guidelines on ED treatment [1]. However, most clinical studies tended to focus on the linear correlation between the intervention methods and the results, therefore ignoring the comprehensive synergistic effect of acupuncture as a complex intervention method. Acupoints can effectively regulate the flow of qi, which results in more qi being brought to the body parts or organs where it is insufficient. If there is too much qi in a region, acupuncture at the corresponding acupoints can also release the excess qi, thus maintaining the balance of Yin and Yang in the body. The regulation of ED using acupuncture has the following objectives: to alleviate the local symptoms of the patients, such as erectile weakness and difficulty in maintaining an erection, to address the overall contributing symptoms, such as fatigue, insomnia, low appetite, and constipation, to identify the syndrome type in the patients according to tongue diagnosis and pulse diagnosis, and to select suitable acupoints for treatment. Therefore, acupuncture can affect the functions of multiple organs or systems working together rather than simply affecting only one body part, the penis [27], which also conforms to the integrated and holistic viewpoint of TCM [28]. Acupuncture works by stimulating various points along the meridians to correct disorders and relieve symptoms without the use of drugs. None of the above four studies mentioned the occurrence of any side effects, except for two cases of premature ejaculation. However, how premature ejaculation occurs remains unclear. Acupuncture is known to be safe, relatively free of side effects, and without adverse physiological impact [29]. Acupuncture may even be cheaper than traditional treatments for some patients, thus making it a viable option for treating ED [30]. The combined application of acupuncture with PDE5Is has also achieved initial results in certain basic studies. Huang et al. showed pharmacokinetic results, demonstrating that low-frequency EA may elevate sildenafil (10 mg/kg, i.v.) concentration in rat plasma, whereas pharmacodynamic investigation revealed that the combined treatment of sildenafil and low-frequency EA enhanced penile circulation in rats [31]. These studies provide evidence for the efficacy of treating ED using acupuncture combined with PDE5Is.

#### 4.1.1. Position and Meridian

Acupuncture, which involves the insertion of needles into specific acupoints, is an ancient alternative therapeutic method to treat various conditions and diseases, including ED. The main acupuncture points used in this review were located on the extremities and abdomen (Figure 2). These points, though sometimes located on the extremities rather than the organs, may regulate some symptoms of the whole body via the action of meridian circulation [32]. For instance, the stimulation of the acupoints on the wrist, such as Nei Guan (PC6), sends afferent discharges to the neurons, inhibits sympathetic output, and decreases the cardiac demand for oxygen [33]. From Figure 2, selecting acupoints from the kidney meridian of the foot-shaoyin, the ren meridian, and back-shu points is commonly used for treating ED. The most frequent acupuncture point used in this review was Guan Yuan (CV4), which is located on the abdomen. The stimulation of this point has been shown to spread to the front of the penis or perineum during treatment [34]. Unlike neuroanatomy, TCM works via distal acupoint selection below the elbow and knee. TCM is a basic method of acupuncture prescription and acupoint selection, which embodies the idea of acupuncture and moxibustion based on syndrome differentiation. In this specific application, it is advisable to utilize not only the meridians of the diseased viscera but also the same-name meridians for the treatment. For example, TCM ascribes ED lesions to issues in the kidney, spleen, or heart meridian. Although the meridians were created based on empiric observations, scientific studies continue to shed light on the complex neurophysiologic mechanisms behind their use in acupuncture [32]. Under the basic principle of distal acupoint selection, Tai Xi (KI3), Zhao Hai (KI6), Nei Guan (PC6), Shen Men (HT7), San Yinjiao (SP6), etc., were selected because of their related meridians. At the same time, the selection of Guan Yuan (CV4), Qi Hai (CV6), and Zhong Ji (CV3) based on the local acupoint selection method of TCM was also reflected.

For the selection of the above methods of acupoint selection, moxibustion is also applicable, which utilizes the warm effect of moxibustion fire to play the dual role of medicine and warmth [35]. The belly button near the abdominal cavity and pelvic area has a wealth of nerve vascular distribution to the bladder. Moxibustion on the ren meridian acupoints, such as guan yuan and qi hai, can act on the nearby plexus to stimulate the penis erection of the cavernous nerve plexus nerve and the prostate and bladder nerves, thus improving urination and penile erectile function. In clinical practice, moxibustion is often combined with other therapies to treat ED. An RCT showed that moxibustion combined with TCM can effectively reduce the IIEF 5 score of ED patients [36].

Although TCM treatment methods were applied in the above four studies, the selection of acupoints was not based on TCM syndrome differentiation. Liu et al. analyzed the acupuncture treatments for ED in 130 classical medical books to summarize the principle of acupuncture for this disease. The results indicated that the characteristics of selecting the acupoints were according to the channels and different syndromes [37]. It is similar to the rules of acupoint selection in this review. However, TCM emphasizes distinguishing the cold and heat of a disease before commencing the treatment and then selecting the corresponding treatment methods and acupoints, which was not reflected in this article and deviated from TCM diagnostic methods.

#### 4.1.2. Intervention

According to the results, the acupuncture courses ranged from 1 to 6 weeks, with a total of 8 to 20 treatments, with each treatment lasting 10, 20, or 30 minutes. An important factor affecting the curative effect is the duration of needle retention. From the point of view of the dose–effect relationship between acupuncture volume and acupuncture effect, the duration of acupuncture retention is an important “dose” for obtaining the acupuncture effect. To a certain extent, there is a positive correlation between the duration of acupuncture retention and the amount of stimulation achieved [38]. The amount of stimulation is closely related to the therapeutic effect on clinical diseases, and the duration of acupuncture retention is very important for the effectiveness of the treatment. However, according to Lin et al., if the needle is kept for a long time blindly, it will not only fail to achieve the desired effect but also produce malignant stimulation, thus reducing the efficacy and even producing adverse reactions [38]. In contrast, if the needle retention time is too short, the optimum stimulation for treating the disease will not be achieved. Either way, it can be difficult to meet the needs of clinical treatment of these conditions. At present, it is generally believed that for central nervous diseases, because of the depth and severity of these conditions, the long-term retention of needles can enhance the amount of acupuncture stimulation. Thus, the acupuncture effect can be gradually accumulated and reach its peak, achieving the maximum amount of stimulation [39]. A long treatment period may be required. From the perspective of TCM, the time and course of acupuncture depends on the severity of the disease, and a shorter period of stimulation and course of treatment may be more suitable for relatively minor functional diseases. Therefore, functional ED caused by central factors seems to fall in between minor and major diseases. The TCM syndrome type of ED and the presence or absence of organic damage, as well as the patient's own constitution, age, and other factors result in varying recommendations when it comes to optimal stimulation time, course of treatment, frequency, and other therapeutic considerations. So far, there is no unified standard, and there are few studies on the relevant mechanisms [40].

EA effectively controls stimulation instead of a manual needle, thus saving personal effort. Generally, EA is combined with ordinary acupuncture, and sometimes electric stimulation is performed at two or more points. Huang et al. studied the effects of EA stimulation at the Guan Yuan (CV4) and Zhong Ji (CV3) acupoints on the mating behavior of sexually experienced male rats. The results showed that the EA of 2 Hz intensity at 1.5 mA (30 min/d, five consecutive days) resulted in longer ejaculation latency. Moreover, the serum 5-hydroxytryptamine (5-HT) and luteinizing hormone (LH) levels of the treated rats were higher than those of the other groups. Therefore, low-frequency EA could effectively improve the sexual behavior of the rats [41]. The choice of TCM acupuncture is not limited to EA. The commonly used techniques also include warm acupuncture and fire acupuncture, which are combined with specific acupoints. In the Liu et al. study, when compared with the control group who used conventional acupuncture, the treatment group subjected to warm needling moxibustion showed higher efficacy and more significantly improved IIEF 5 scores [42]. However, these results revealed there was little significant difference in efficacy between EA and non-EA treatments. Because of the lack of relative clinical studies and limitations of personal situations, treatment course, doctors' levels, acupoints, and other factors, there is no indication as to which technique is better for treating ED.

#### 4.1.3. Evaluation of Therapeutic Efficiency

Acupuncture treatment is a process of overall adjustment and personalization, which is reflected in the improvement of the patients' systemic symptoms. This improvement is one of the advantages of acupuncture. Therefore, it is necessary to include TCM symptom scores and characteristics in the outcome index to observe the changes in concomitant symptoms other than poor erection. Although there is still no definite conclusion on the effect of acupuncture on sex hormone levels, testosterone (T) can be used as an observation indicator before and after treatment because of its potential effect on male sexual function. Meanwhile, the erection angle and success rate of sexual intercourse should not be ignored. In the past, the attention to sexual dysfunction was mostly limited to men [43]. With the improvement in the population's health awareness and the abundance of diagnosis and treatment methods, sexual satisfaction of partners has also now been applied in the efficacy evaluation of ED [44]. ED is a male sexual dysfunction. However, it can also have an impact on the female partner's sexual experience and their quality of life. ED can cause serious negative effects [45], and women are also concerned about this problem. Their sexual needs may give men psychological pressure and even cause family conflicts. Therefore, the role of the female partners in the diagnosis and treatment of ED cannot be ignored [46]. The partners of those under treatment may notice an improvement in their mate's confidence levels and mood, thereby affecting the marital relationship both inside and outside the bedroom [47]. Since ED involves emotional factors and most studies tend to be psychological, the relevant scales also need to be enriched. It is recommended by the guidelines to use the erectile hardness score or the assessment of penile rigidity in practice and in clinical trials research [6, 48].

### 4.2. Possible Mechanisms

#### 4.2.1. Acupuncture May Improve Regulation of the Hypothalamus

Based on the above results, functional ED was found to be effectively treated using acupuncture, especially in the aspect of psychological symptoms. Evidence shows that more than 50% of patients with ED suffer from depression, with the degree of depression linked to the severity of ED [49, 50]. The rates of depression drop drastically as ED becomes effectively treated [51]. Depression is closely related to the hypothalamic–pituitary–adrenal (HPA) axis [52]. When the HPA axis is hyperfunctional, the prevalence of depression is significantly increased [28]. Lee et al. reported that acupuncture at Nei Guan (PC6) significantly reduced CORT-induced anxiety and depression behaviors in rats and increased the expression of neuropeptide Y in the hypothalamus [53]. Many *in vivo* studies have shown that neuropeptides are critical for the central control of male sexuality and are involved in pain relief mechanisms after acupuncture [54–56]. This finding indicates that acupuncture may alleviate anxiety and depression in the patients by regulating the HPA axis, thus effectively treating ED. Another study showed that with low-frequency EA, serum 5-HT levels and sexual behavior improved in rats [41]. Furthermore, Hagemann et al. [57] applied positron emission tomography to study the brain structure and metabolism of psychological ED and found that glucose metabolism in the bilateral hypothalamus increased significantly in healthy volunteers after receiving audio–visual stimulation. Nonetheless, glucose metabolism in the bilateral hypothalamus did not increase significantly in patients with psychological ED after receiving the same stimulation. Dong et al. [58] confirmed in their studies that the efficacy of acupuncture is closely related to blood flow, oxygen metabolism, and glucose metabolism in certain regions of the brain. This result also indicates that some functional areas in the hypothalamus may be abnormal in patients with ED and that acupuncture can improve their regulatory activities by enhancing brain metabolism.

#### 4.2.2. Effect of Acupuncture on Reproductive Hormone Levels

The changes in male sex hormone levels are most closely related to sexual function [59]. *T* indirectly promotes penile erection by enhancing sexual desire and arousal and plays an important role in maintaining the normal structure of penile erection [60]. There were no significant alterations in the levels of hormones, such as adrenocorticotropic hormone (ACTH), antidiuretic hormone (ADH), follicle stimulating hormone, LH, prolactin (PRL), and *T* during and after the treatment sessions from Kho [20]. Because of the lack of included literature, the relevant results may be unrepresentative. Zhang et al. [61] observed 60 patients with male impotency who exhibited ED before and after acupuncture. The investigators measured serum *T*, estradiol (E2), and PRL and found that after treatment, serum *T* level increased, E2 and PRL content decreased, and normal sexual behavior was maintained in the patients with ED. This finding suggests that acupuncture can effectively correct disorders related to serum hormone levels in patients with ED, and therefore, improve the clinical symptoms.

#### 4.2.3. Acupuncture May Affect the Local Nerves

The penis is composed of arterioles and capillaries, blood filled sinuses, and smooth muscles. Normal erection is initiated through external stimuli via somatic and autonomic pathways [62]. The autonomic nerve originates from an important branch of the pelvic plexus, i.e., the cavernous nerve. The autonomic nerve contains sympathetic and parasympathetic nerve fibers. The parasympathetic nerve postganglionic fibers are distributed in the penile vascular smooth muscle, cavernous smooth muscle, and cavernous sinus small beampost smooth muscle, which are the main nerve fibers involved in penile erection [63]. Sympathetic postganglial fibers are distributed along the parasympathetic fibers, and their function is to maintain the status of normal penile flaccidity, return to a penile flaccidity after erection, and promote the psychological erection. The somatic nerve originates from the pudendal nerves, whose sensory branch senses the penis and perineum and transmits information to the reproductive center of the spinal cord to participate in reflex erection, and the motor branch innervates the skeletal muscle of the perineum. The spinal erectile center is located in the T12-L1 segment, and the reflex erectile center is located in the S2–S4 segment. The acupuncture of the spinal erectile center with the ganglial segment of the Ci Liao (BL32), Zhong Ji (CV3), Zhi Bian (BL54), and Da He (KI12) can significantly improve the spinal erectile center excitability and improve the erectile state. For example, evidence shows that acupuncture into Zhong Ji (CV3) can also obtain a sensation radiating toward the perineum and the lower abdomen, thus achieving a therapeutic effect for genitourinary diseases [41]. The acupoints were inferred, and it was observed that the inferior nerve derived from T11-L1 in the abdominal region may be effective in the treatment of urinary tract diseases and play a regulatory role in the prostate [64]. The stimulation of the perineal striated muscle by the pudendal nerves can improve the rigidity of the penile tissue [65, 66], and acupuncture can have an effect on pelvic nerve outflow [67].

#### 4.2.4. Acupuncture May Affect the Release of Nitric Oxide in the Blood Vessels of the Penis

Nitric oxide synthase (NOS) and nitric oxide-cyclophosphoguanosine (NO-CGMP) signaling pathways play key roles in achieving penile erection. This result suggests that changes in NOS and NO-CGMP in the penile tissue may affect penile erectile function. Acupuncture may modulate the release of NO and some neuropeptides involved in the process of erection [17, 68, 69]. Yang et al. [70] studied the effects of moxibustion on diabetic ED rats and found that acupuncture could significantly improve the levels of NOS and NO-CGMP in the penis tissue, thus improving their erectile function. Previous studies also confirmed that acupuncture can affect pelvic nerve outflow [67]. A spinal reflex involving NO and modulated by various brain centers, such as the hypothalamus and periaqueductal gray, also plays a role, but it is unclear if acupuncture needling is sufficiently local to influence the release of NO in the appropriate vessels [71, 72].

## 5. Limitations

In this review, in strict accordance with the retrieval strategy, only 4 pieces of English literature were included. Some studies in other languages were not covered owing to language barriers. Hence, the small sample size and the low quality of the trials might have led to a bias. However, the purpose of this study was to review the possible mechanisms of acupuncture treatment for ED and to analyze the corresponding treatments in terms of TCM characteristics and advantages. The inadequate evidence and the high heterogeneity of the studies might have led to an insufficient understanding of the related mechanisms. It is difficult to determine the efficacy and safety, although the above four studies have consistently shown that acupuncture has high efficacy [17, 73].

## 6. Conclusion

In the treatment of ED, the selection of the acupoints is focused on ren meridians and kidney meridians, often combining the acupoints at the distal ends of the extremities and abdomen. The results of the present research show that acupuncture is effective in the treatment of ED, especially functional ED, and conforms to the guidelines for providing comprehensive treatment but is limited by insufficient evidence. Hence, its effectiveness and safety need to be further verified, and the specific mechanism needs to be further explored. There is no clear standard for the time and course of acupuncture treatment for ED, and the choice of EA has not been unified.

In conclusion, this review will help the clinicians in treating ED and provide potential evidence and trends for future research. Patients with ED may also benefit from potential alternative interventions.

## Figures and Tables

**Figure 1:** Flow chart of the study search.

**Figure 2:** The location and distribution of the acupuncture points. The red, blue, green, and yellow circles represent the acupoints selected by Engelhardt et al., Aydin et al., Kho et al., and Yaman et al., respectively.

**Table 1:** PubMed search strategy.

	No. search item
#1	Acupuncture (title/abstract)
#2	Acupuncture treatment (title/abstract)
#3	Electroacupuncture (title/abstract)
#4	Acupuncture therapy (title/abstract)
#5	Fire needling (title/abstract)
#6	Scalp acupuncture (title/abstract)
#7	Ear acupuncture (title/abstract)
#8	Or/#1– #7
#9	Erectile dysfunction (title/abstract)
#10	Impotence (title/abstract)
#11	Erection failure (title/abstract)
#12	Penis erection (title/abstract)
#13	Male sexual dysfunction (title/abstract)
#14	Or/#9–#13
#15	Clinical trial (publication type)
#16	Clinical article (publication type)
#17	Clinical study (publication type)
#18	Controlled study (publication type)
#19	Randomized controlled trial (publication type)
#20	Placebo (publication type)
#21	Or/#15–#20
#20	#8 and #14 and #21

**Table 2:** Summary of the included studies.

References	Study design	Type	Sample	Acupuncture points	Intervention	Outcome	Effective rate	Adverse event
Engelhardt et al. [18]	RCT	Psychogenic	10	Zhao Hai (KI6), Shu fu (KI27), Guan Yuan (CV4), Qi Hai (CV6), Shen Shu (BL23), Wan Gu (SI4), San Yinjiao (SP6)	AC, 20 min 1–2/week for 5–20 sessions	Self-sexual activity satisfaction IIEF 5	68%	None

Aydin et al. [19]	RCT	Nonorganic	15	Qi Chong (ST30), Zu Sanli (ST36), Zhao Hai (KI6), Guan Yuan (CV4), Qi Hai (CV6)	EA, 20 min 2/week for 6 weeks	Self-sexual activity	60%	None

Kho et al. [20]	UCT	9 psychogenic 4 organic 3 discontinued	16	Guan Yuan (CV4), Bai Hui (GV20), San Yinjiao (SP6), tai Xi (KI3), Shen Men (HT7)	AC + EA, 30 min 2/week for 4 weeks	Self-sexual activity partner's activity satisfaction profiles of hormones	54%	Not mentioned

Yaman et al. [21]	UCT	Psychogenic	29	Ci Liao (BL32), Da Dun (LR1), Yin Lian (LR11), Nei Guan (PC6), tiao Kou (ST38), Qu Gu (CV2), Bai Hui (GV20)	AC, 10–20 min total 10 sessions 3/week for week 1 2/week in the following weeks	Self-sexual activity	69%	Two patients had premature ejaculation

AC: acupuncture, EA: electric acupuncture, UCT: uncontrolled clinical trial, and RCT: randomized controlled trial.

## Data Availability

Specific study data are available from the corresponding author upon request.
